RETRACTED

# Exploration of the Effect of Icariin on Nude Mice with Lung Cancer Bone Metastasis via the OPG/RANKL/RANK System

**DOI:** 10.1155/2022/2011625

**Published:** 2022-05-28

**Authors:** Zhao Ruilian, Gao Ying, Shen Hongmei, Guo Lihua

**Affiliations:** ^1^Department of Integrated Traditional and Western Medicine, Tumor Hospital of Yunnan Province, The Third Affiliated Hospital of Kunming Medical College, Kunming, Yunnan 650118, China; ^2^College of Clinical Medicine, Nanjing University of Traditional Chinese Medicine, Nanjing, Jiangsu 210000, China; ^3^Department of Physiatry, The Second People's Hospital of Kunming, Kunming, Yunnan 650000, China; ^4^Traditional Chinese Medicine Hospital of Yunnan Province, Kunming, Yunnan 650000, China

## Abstract

Epimedium is a traditional Chinese medicine that is most commonly prescribed by practitioners of Chinese medicine for the clinical treatment of malignant tumor bone metastasis. The main component of Epimedium is icariin (ICA). Studies have shown that ICA inhibits bone resorption of osteoclasts through the OPG/RANKL/RANK signaling pathway. Osteoclasts are the only cells in the body that have a bone-destroying capability. The OPG/RANKL/RANK system consists of cytokines that play major roles in osteoclast formation. Therefore, our study selected the OPG/RANKL/RANK system as the research target to investigate the effect of ICA on nude mice with lung cancer bone metastasis. We established the model of bone metastasis in nude mice, intervened the model with icariin and zoledronic acid, and detected the levels of OPG and RANKL by ELISA and western blot. The results showed that ICA had a significant inhibitory effect on bone metastases in nude mice. ICA achieved its antibone metastasis effect in nude mice with lung cancer via inhibiting RANKL expression and simultaneously increasing OPG expression. ICA not only alleviated osteolytic bone destruction caused by bone metastases, but it also reduced weight loss in tumor-bearing nude mice at the late stage of the experiment. The role of ICA in preventing bone metastasis of lung cancer merits further investigation.

## 1. Introduction

The predilection sites for metastases from lung cancer are the bones [1]. Bone metastasis causes a series of complications such as severe pain, pathological fracture, fatal hypercalcemia, spinal cord compression, and other nerve compression symptoms, which seriously affect the quality of life of the patients [2–4]. Currently, the drugs used in clinical practice to prevent and treat bone metastasis are mainly bisphosphonates [5–7]. These drugs not only display inhibitory effects toward bone destruction but also have antitumor effects. However, long-term use of bisphosphonates may lead to side effects (such as anemia, thrombocytopenia, bone pain, and renal functional impairment), which limits the application of the drugs to a certain extent [8–10].

RETRACTED

Epimedium (Yin Yang Huo) is a Chinese herbal medicine that is commonly used in clinical practice for bone injury [11, 12]. Icariin (ICA) is one of the main components of Epimedium extract. In recent years, a number of studies focusing on various bone injuries in animal models of experimental osteoporosis have confirmed the direct effects of Epimedium [13–16] or icariin on the skeletal system and the effects of Epimedium on the expression of bone-related proteins and genes [17–19]. Early in 1985, some Chinese researchers found that Epimedium injection can significantly promote the growth of chicken embryo femur and the synthesis of proteoglycan in vitro, suggesting that Epimedium has a direct effect on the bone system. The results of systematic review and meta-analysis demonstrated that ovariectomized rats treated with icariin had significantly higher bone mineral density (femur and lumbar spine) and lower bone turnover markers (serum alkaline phosphatase and osteocalcin) compared with the ovariectomized control group [20]. Some studies have showed that icariin can prevent overall progression of chronic high-dose alcohol-induced osteopenia in a rat model, in a dose-dependent manner. Icariin promotes bone formation and inhibits bone loss and effectively restores bone structure and strength in chronic high-dose alcohol-induced osteopenic rats. Bone metabolism reversal is evidenced by increased BV/TV, BMD, MAR, percent trabecular area, and biomechanical properties and elevated [21]. The researchers used New Zealand rabbits as models which were immunized with antigen-induced arthritis (AIA) and treated with icariin. Histological analysis and TEM sections of cartilage in the ICA-treated group showed a low level of chondrocyte destruction. Micro-CT analysis showed that the bone mineral density value and bone structural level in ICA-treated rabbits were significantly higher compared with those in the AIA group. Immunohistochemistry and real-time PCR analysis showed that icariin treatment reduced RANKL expression and enhanced OPG expression levels, as compared to the AIA group. These data indicate that ICA suppresses articular bone loss and prevents joint destruction. This study also determined that ICA regulated articular bone loss in part by regulating RANKL and OPG expression [22].

In addition, the antitumor mechanisms of Epimedium have been explored in many experimental studies. Research demonstrated that ICA has the potential to upregulate LMP/TAP-related molecules and induce the expression of MHC-I, which increases the immune surveillance and keeps cancer in remission. ICA showed an antitumor effect both in vitro and in vivo and may be an effective antigen adjuvant for cancer treatment by enhancing tumor-specific immunity [23]. Some researchers found that icariin can suppress tumor growth and enhance the antitumor activity of 5-FU in CRC by inhibiting NF-*κ*B activity. The antitumor activity of icariin is implicated in the suppression of NF-*κ*B activity and consequent downregulation of the gene products regulated by NF-*κ*B [24].

RETRACTED

However, there are few reports on the experimental study of icariin for the antibone metastasis of malignant tumors. Many studies have shown that osteoclasts are the only cells that can destroy bone in vivo. OPG/RANKL/RANK system is a cytokine that plays a major role in the formation of osteoclasts. Therefore, the present study established a nude mice model of lung cancer bone metastasis as the research objective and explored the mechanisms of action of ICA in the nude mice model of lung cancer bone metastasis based on a series of cytokines that play major roles in osteoclast formation (namely, osteoprotegerin (OPG)/receptor activator of nuclear factor kappa-*Β* ligand (RANKL)/receptor activator of nuclear factor kappa-*Β* (RANK)).

## 2. Materials and Methods

### 2.1. Experimental Animals and Cells

Specific pathogen-free (SPF) grade nude mice, 4-6 weeks of age and weighing approximately 19-20 g, were purchased from Beijing Hua Fukang Biotechnology Co., Ltd. and maintained in the Cancer Research Institute of Yunnan Cancer Hospital. SPC-A-1 lung cancer cells were purchased from the cell bank of Chinese Academy of Science, Shanghai, and subcultured in the Cancer Research Institute of Yunnan Cancer Hospital.

### 2.2. Cell Culture

SPC-A-1 lung cancer cells were cultured in high-glucose Dulbecco's Modified Eagle's Medium (DMEM, Sigma, USA) supplemented with 10% fetal bovine serum (FBS, Sigma) and 1% penicillin/streptomycin (Sigma) under standard conditions (37°C, 5% CO_2_, and saturated humidity). The cells were passaged when cell viability exceeded 90%, and the cell adherence rate reached 80%-90%. To passage the cells, the cells were digested with trypsin. Cells in the logarithmic growth phase at a density of 80-90% were collected for future assays.

### 2.3. Establishment of the Animal Model

A total of 24 nude mice were divided into 4 groups using the random number method (6 mice per group). The care of the animals involved in the experiments and procedures was conducted in conformity with the guidelines on the Administration of Lab Animals and the guidelines on the Humane Treatment of Laboratory Animals (MOST 2006a). This study was approved by the Animal Care and Use Committee of Kunming Medical College (Kunming, China).

RETRACTED

The 4 groups included the blank bone metastasis model group (NS), the ICA (CAS: 489-32-7, PLC ≥ 98%; Sichuan Victory Biological Technology Co., Ltd., China) 20 mg/kg + bone metastasis group (ICA20), the ICA 10 mg/kg + bone metastasis group (ICA10), and the zoledronic acid (H20140218, Swiss Novartis Pharmaceutical Co., Ltd.) + bone metastasis group (ZOL). Cells in the logarithmic growth phase at a density of 80-90% were used to construct the animal model. One day before the cells were collected, the culture medium was removed and replaced with fresh medium. Prior to trypsin digestion, 7 large flasks of cells were examined under a microscope (Olympus, Japan) to confirm the absence of contamination. After trypsinization, the cells were collected. The collected cells were washed three times with precooled normal saline to completely remove the serum. Subsequently, the cell pellets were diluted in normal saline to the desired concentration. Each mouse was inoculated with 3 × 10^6^ cells, and the inoculation volume was 30 *μ*L/mouse. After the cells were digested, counted, and diluted, the centrifuge tubes containing the cell suspension were placed on ice, which reduced cell metabolism and ensured cell viability.

Prior to inoculation, the cells in the cell suspension were thoroughly dispersed with a Pasteur pipette, which prevented the reduction of the cell survival rate caused by cell clustering. At the time of cell inoculation, the mice were immobilized using restrainers. The cells were then inoculated using disposable insulin syringes.

The conditions of the mice were observed daily after inoculation of the cells, including food intake, water intake, hair color, mental state, tumor metastasis, and tumor growth. In addition, all groups of nude mice were weighed before establishment of the bone metastasis model, on the 3rd, 10th, and 17th days after establishment of the bone metastasis model and before sacrifice of the mice. The details of the body weight changes in all groups of mice were recorded.

### 2.4. Mode of Administration

ICA (20 mg/bottle) was first dissolved in 200 *μ*L of dimethyl sulfoxide (DMSO) and then adjusted to the desired concentrations with normal saline (20 mg/kg and 10 mg/kg group). The prepared ICA solution was stored at 4°C for future assays. The dose administered to the mice was calculated according to the following formula: 9.1 × mg/kg. Since the average body weight of the mice was 20 g, the actual doses administered were 3.64 mg/mouse (ICA20) and 1.82 mg/mouse (ICA10). Both groups of mice received intragastric administration of ICA on the 3rd day after inoculation of tumor cells. Thereafter, ICA was administered once daily (0.1 mL) for a total of 20 doses.

RETRACTED

Zoledronic acid (4 mg/bottle) was first dissolved in 5 mL of sterile saline and then diluted to 4 *μ*g/mL with 1000 mL of 0.9% normal saline. The normal dosage for humans is 4 mg/50 kg (i.e., 0.08 mg/kg). Therefore, the dose administered to the mice would be 0.728 mg/kg according to the formula 9.1 × mg/kg. Since the average body weight of the mice was 20 g and the volume of the intraperitoneal injection was 0.2 mL, the content of zoledronic acid would be 0.4 *μ*g. The mice received an intraperitoneal injection of zoledronic acid on the 3rd day after inoculation of tumor cells. Thereafter, zoledronic acid was injected once every other day (0.2 mL) for a total of 10 doses.

### 2.5. Specimen Collection

All sacrificed mice were dissected. The mouse skull, spine, ribs, limb bones, scapulae, and pelvises were examined by the naked eye for the formation of bone metastases. In addition, the number of bone metastases was recorded.

After the bone metastases and the suspected bone metastases were removed, tumor size was measured. Specifically, the longest and the shortest axes of the tumors were measured using an electronic Vernier caliper.

Mouse blood was extracted from the eyeballs, placed at room temperature (RT) for 30 min, and then centrifuged at 3000 r/min for 5 min. The sera was transferred to 1.5-mL cryotubes and stored at -80°C in an ultra-low temperature freezer.

The collected tumors were photographed with a digital camera. A portion of the tumors was quickly frozen in liquid nitrogen for western blot analysis, while another portion was fixed in formalin for pathological examination.

### 2.6. Enzyme-Linked Immunosorbent Assay (ELISA)

ELISA was used to analyze the levels of RANKL and OPG in serum samples of the nude mice. In the pre-experiments, standard curves were generated based on the standards provided in the kit. In addition, two randomly selected serum samples were diluted to obtain a gradient to determine the optimal dilution ratios for the analysis of the serum samples and standard curves. Standard curves were also plotted in the formal experiment. All serum samples were diluted according to the ratio determined in the pre-experiment. The data were analyzed using a microplate reader (Thermo Scientific, USA). All serum samples were diluted according to the ratio determined in the pre-experiment. Sample analysis was performed in single-wells.

### 2.7. Western Blot

Total protein was extracted from various groups of tissue specimens. First, radioimmunoprecipitation assay (RIPA) lysis buffer was mixed thoroughly with phenylmethanesulfonyl fluoride (PMSF) at a volume ratio of 100 : 1. The mixture was placed on ice for future use. Subsequently, the weighed tissue specimens were cut into small pieces using disinfected scissors and transferred to the bottom of the homogenizer. The prepared lysis buffer was then added at a ratio of 1 part lysis buffer to 1 gram of tissue. After addition of the lysis buffer, the tissue specimens were homogenized at high speed for several minutes on ice in an attempt to completely break down the tissues. The liquid in the homogenizer was transferred to Eppendorf (EP) tubes, further lysed on ice for 30 min, and then centrifuged at 4°C and 1200 r for 30 min. The resulting supernatants were the total protein solution. The supernatants were collected, aliquoted, and stored at -80°C. The supernatants were subjected to protein quantification by the Bradford method using bovine serum albumin (BSA) as the standard. Glyceraldehyde 3-phosphate dehydrogenase (GAPDH) was used as an internal reference protein. Protein samples (20 *μ*g each) were separated by sodium dodecyl sulfate polyacrylamide gel electrophoresis (SDS-PAGE) on a 10% gel, transferred to nitrocellulose membranes (100 V, 1 h), blocked in blocking solution at 37°C for 1 h, and incubated with primary antibodies at 4°C overnight. Moreover, another membrane was incubated with Tris-buffered saline-Tween-20 (TBS-T) solution containing no primary antibody, which served as the negative control. After repeated washing, the membranes were incubated with alkaline phosphatase (AP)-labeled anti-IgG antibody at RT for 1 h with gentle shaking. After washing, the expressions of RANKL and OPG were examined by western blotting. The absorbance (A) value of each band was determined by image analysis and quantitatively analyzed.

RETRACTED

### 2.8. Pathological Hematoxylin and Eosin (HE) Staining

Paraffin sections were prepared from tissues fixed in 10% neutral formalin solution via the following steps: fixation, dehydration, clearing, infiltration, embedding, and sectioning. After the tissue sections were stained with HE and mounted in neutral resin, the histomorphological characteristics of the mouse bone metastases were examined under a microscope.

### 2.9. Statistical Analysis

The data in the present study were analyzed using SPSS 21.0 software. The means of multiple samples were subjected to significance testing using one-way analysis of variance (ANOVA). Nonparametric statistical analysis of quantitative survival data was conducted to compare the survival rates of the mice. A *p* value of less than 0.05 was considered statistically significant.

## 3. Results

### 3.1. General Condition of the Animals

The survival of mice in each group was observed after the establishment of the model. During the experimental period, there were 2 deaths in the NS group and 1 death in the ICA10 group. None of the mice in the ZOL group and ICA20 group died. However, there was no statistically significant difference in the mortality rate among the groups of mice (*p* > 0.05).

Body weight changed in various groups of mice during the experimental period. Before construction of the bone metastasis model, there was no significant difference in the average body weight between the groups of mice (*p* > 0.05). On the 3rd day after the establishment of the model (i.e., at the start of drug administration), none of the mouse groups exhibited a significant change in average body weight. In addition, there was no significant difference in the average body weight among the groups (*p* > 0.05). On the 10th day after establishment of the model (i.e., after 1 week of drug administration), all groups of mice showed varying degrees of average body weight loss. However, there was still no significant difference in average body weight among the groups (*p* < 0.05). On the 17th day after establishment of the model (i.e., after 2 weeks of drug administration), all groups of mice continued to show a decrease in average body weight. The average weight loss in the NS group was not significantly different from that in the ZOL group and ICA10 group (*p* > 0.05). However, a significant difference in the average weight loss was detected between the NS group and ICA20 group (*p* < 0.05). There was no significant difference between all the other groups. Before the mice were sacrificed (i.e., after 3 weeks of drug administration), all groups of mice continued to show a decline in average body weight. In addition, mouse activity, food intake, and water intake also decreased. Two mice in the NS group and one mouse in the ICA10 group died. The average weight loss in the NS group was not significantly different from that in the ZOL group and ICA10 group (*p* > 0.05). However, a significant difference in average weight loss was detected between the NS group and ICA20 group (*p* < 0.05) and between the ZOL group and ICA20 group (*p* < 0.05) (Table 1).

### 3.2. Tumor Growth Status

Femoral cavity injection resulted in a tumorigenesis rate of 100% in all groups of mice. However, no distant bone metastasis and metastasis to other organs occurred. After the mice were sacrificed, the femur metastases were removed, and the volume and weight of the metastatic tumors were measured (Figure 1(a)). The mean tumor volume and weight were significantly decreased in the ICA20 group in comparison to the NS, ZOL, and the ICA10 groups (*p* < 0.05). In contrast, there was no significant difference in tumor volume and weight among the other groups (*p* > 0.05) (Figures 1(b) and 1(c)).

RETRACTED

### 3.3. Pathological Examination of Mouse Bone Metastases

One specimen of bone metastases was randomly selected from each group for pathological examination. After fixation and decalcification, the specimens were embedded in paraffin and sectioned. HE staining was performed to examine the effect of tumors on bone injury (Figure 2). The results showed that in the NS group, lung cancer cells caused apparent bone destruction. In addition, the infiltration of a large number of irregular tumor cells was observed in the bone cortex and medullary cavity. The tumor cells had enlarged nuclei and displayed apparent atypia. Certain amounts of tumor cells were observed in the medullary cavity of the mice in the ZOL and ICA10 groups. However, the ZOL and ICA10 groups displayed lower degrees of bone destruction and trabecular bone destruction in comparison to the NS group. In the ICA20 group, a certain number of tumor cells were present in the medullary cavity. Bone destruction and trabecular bone destruction were less severe in the ICA20 group than in the NS, ZOL, and ICA10 groups.

### 3.4. ELISA Analysis of RANKL and OPG Levels in Mouse Serum

The ELISA results are shown in Figure 3. Compared with the NS group, the serum OPG and RANKL levels and OPG/RANKL ratio were significantly increased in all other groups (*p* < 0.05). The serum OPG levels were significantly increased in the ICA10 group in comparison to the ZOL group. However, there was no significant difference in serum RANKL content between the ZOL group and ICA10 group (*p* > 0.05). The serum OPG and RANKL levels and OPG/RANKL ratio were significantly increased in the ICA20 group in comparison to the ZOL group (*p* < 0.05).

### 3.5. Western Blot Analysis of RANKL and OPG Expression in Bone Metastases

Two specimens were randomly selected from each group and subjected to western blot analysis. The results are shown in Figures 4(a)–4(c). Compared with the NS group, all other groups showed significantly increased expression levels of OPG and RANKL proteins and a significantly elevated OPG/RANKL ratio in the bone metastases (*p* < 0.05). Compared with the ZOL group, the expression of OPG was significantly increased in the ICA10 group (*p* < 0.05). However, there was no significant difference in RANKL expression between the ZOL group and ICA10 group (*p* > 0.05). The serum OPG and RANKL levels and OPG/RANKL ratio were significantly increased in the ICA20 group in comparison to the ZOL group (*p* < 0.05). The results were basically consistent with the expression levels of OPG and RANKL in serum.

RETRACTED

## 4. Discussion

Epimedium is a traditional Chinese medicine that is most commonly prescribed by practitioners of Chinese medicine for the clinical treatment of malignant tumor bone metastasis. The main component of Epimedium is ICA [25]. To date, a large number of studies have described the intervening effect of ICA, the main component of Epimedium, in various animal models of bone injuries (mainly experimental osteoporosis) and various bone-related cells (mainly osteoblasts). Studies have shown that a combination of ICA and stem cells not only improves the osteoporosis-induced bone loss and microstructural destruction of bone tissue in a rat model but also reduces liver and kidney damage in osteoporotic rats [26]. A meta-analysis of the antiosteoporotic effect of ICA showed that ICA has a significant antiosteoporotic effect in ovariectomized rats [27]. In addition, a number of studies have shown that ICA inhibits bone resorption of osteoclasts through the OPG/RANKL/RANK signaling pathway [28].

Osteoclasts are the only cells in the body that have a bone-destroying capability. There is currently no conclusive evidence that tumor cells have the ability to directly destroy bone. The OPG/RANKL/RANK system consists of cytokines that play major roles in osteoclast formation. Osteoclasts originate from the mononuclear macrophage system in hematopoietic tissues. The formation of osteoclasts is regulated by a variety of physicochemical factors. The interaction of RANKL/RANK molecules represents the ultimate common pathway in this process. In the presence of macrophage colony-stimulating factor (M-CSF), osteoclast precursors or osteoclasts contact osteoblasts or bone marrow stromal cells, which allow the binding of RANKL to RANK. Binding of RANKL to RANK stimulates the activation and differentiation of osteoclasts via intracellular signaling pathways. OPG blocks the interaction between RANKL and RANK by binding to RANKL, thereby inhibiting the differentiation of osteoclasts and reducing bone resorption. Therefore, OPG/RANKL/RANK form a trinity system: RANKL on the surface of osteoblasts binds to RANK on the surface of osteoclasts, which promotes the maturation and activation of osteoclasts. In addition, osteoblasts secrete OPG, which binds to RANKL. The binding of OPG/RANKL prevents RANKL from binding to RANK on the surface of osteoclasts and terminates bone resorption, thereby regulating bone resorption and bone formation [29].

The OPG/RANKL/RANK system is closely related to bone destruction caused by malignant tumors [30]. The mechanisms by which tumor metastasis induces bone destruction have been studied [31]. It is currently believed that metastatic tumor cells directly or indirectly activate the differentiation and maturation of osteoclasts and osteoblasts, resulting in tumor-induced osteoclastic and osteogenic bone destruction [32, 33].

RETRACTED

Therefore, the present study selected the OPG/RANKL/RANK system as the research target to investigate the effect of ICA on nude mice with lung cancer bone metastasis. The results showed that ICA had a significant inhibitory effect on bone metastases in nude mice. The tumor volume and weight were reduced in the ICA20 group in comparison to the NS, ZOL, and ICA10 groups. No significant differences were observed in tumors between the ICA10 group and blank group. However, the average tumor volume and tumor weight were increased in the ICA10 group compared with the ZOL group. At the end of the experiment, the extent of weight loss was less pronounced in the ICA20 group in comparison to the NS, ZOL, and ICA10 groups. None of the mice in the ICA20 group had died by the end of the experiment. Moreover, food and water intake were more normal in the ICA20 group compared with the other groups. These results demonstrated that, compared with zoledronic acid, a high dose of ICA not only provided a tumor inhibitory effect but also improved the overall life quality of the nude mice. However, the above effects were not apparent in the low-dose ICA group.

To examine the degree of bone destruction, randomized pathological HE staining of bone metastases was performed in the four groups of specimens. Compared with the NS group, a lower degree of bone destruction was observed in the ICA20, ZOL, and ICA10 groups. The ICA20 group showed the lowest degree of bone destruction. Moreover, tumor cell infiltration was reduced in the ICA20 group in comparison to the other groups. The above results demonstrated that ICA improved the tumor-induced osteolytic destruction of femur bone in nude mice.

In the present study, ELISA and western blot analysis of the OPG/RANKL/RANK system yielded consistent results. The serum and tumor tissue expression of OPG were the highest in the ICA20 group among all the groups. Western blot analysis of the tumor tissues showed that the expression level of RANKL was higher in the ICA20 group than in the ZOL group. However, the ICA20 group showed the lowest OPG/RANKL ratio among all the groups, which was consistent with the lowest degree of bone destruction in the ICA20 group. The effect of low-dose ICA (ICA10 group) on OPG/RANKL/RANK was weaker than that of ZOL. However, OPG expression was still significantly higher in the ICA10 group in comparison to the NS group. In contrast, RANKL expression was significantly lower in the ICA10 group in comparison to the NS group. The above results demonstrated that the inhibitory effect of ICA on lung cancer bone metastasis was no weaker than zoledronic acid. Moreover, compared with zoledronic acid, ICA had an overall inhibitory effect on tumors.

RETRACTED

Recent research has confirmed ICA can regulate bone formation by upregulating the OPG/RANKL expression ratio in human osteoblast cells [34]. ICA could alleviate or lessen the degree of articular cartilage destruction in CIA rats, and its mechanism might be associated with reducing serum levels of RANKL and elevating levels of OPG, thus further decreasing the ratio of RANKL/OPG [35]. ICA could inhibit bone resorption of osteoclasts through regulating the OPG/RANKL signal pathway [36]. Our results are basically consistent with the results obtained by other researchers in experimental studies of the antitumor effect of ICA. Comparing these studies, this study confirmed that ICA can also regulate bone formation by upregulating the OPG/RANKL expression ratio on bone metastases of mice for the first time.

In summary, the results of the present study showed that ICA achieved its antibone metastasis effect in nude mice with lung cancer via inhibiting RANKL expression and simultaneously increasing OPG expression. ICA not only alleviated osteolytic bone destruction caused by bone metastases, but it also reduced weight loss in tumor-bearing nude mice at the late stage of the experiment. The role of ICA in preventing bone metastasis of lung cancer merits further investigation. There is currently no precedent for the use of ICA alone in clinical practice in the form of a traditional Chinese medicine monomer. However, it is often used clinically as an ingredient in compounds in Chinese medicines. Therefore, the antitumor and antibone metastatic effects of ICA in the nude mouse model of lung cancer bone metastasis necessitate further and in-depth pharmacological, toxicological, and mechanistic investigations.

## Figures and Tables

**Figure 1:** Effect of Icariin on xenograft tumor growth. (a) Images of representative tumors excised from mice in each groups. Tumor volume (b) and weight (c) were measured. ∗*p* < 0.05 vs. NS group; #*p* < 0.05 vs. ZOL group. NS: the blank bone metastasis model group; ZOL: the zoledronic acid + bone metastasis group; ICA20: icariin 20 mg/kg + bone metastasis group; ICA10: icariin 10 mg/kg + bone metastasis group.

**Figure 2:** HE staining of tumor in various groups. (a1 and a2) NS group; (b1 and b2) ZOL group; (c1 and c2) ICA10 group; (d1 and d2) ICA20 group. (a1)–(d1) ×4 magnification; (a2)–(d2) ×20 magnification.

RETRACTED

**Figure 3:** Comparison of ELISA analysis of RANKL and OPG levels in different groups. ∗*p* < 0.05 vs. NS group; #*p* < 0.05 vs. ZOL group.

**Figure 4:** Effect of icariin on the protein expressions of OPG/RANKL. (a) The protein expressions of OPG and RANKL were detected by western blot. (b) Gray value analysis of OPG and RANKL. (c) The ratio of OPG/RANKL. ∗*p* < 0.05 vs. NS group; #*p* < 0.05 vs. ZOL group.

**Table 1:** Body weight changes of mice in various groups (g).

Group	D0	D3	D10	D17	D21
NS	19.78 ± 0.53	19.81 ± 0.85	18.75 ± 0.62	17.03 ± 0.52	16.61 ± 0.42
ZOL	19.89 ± 0.78	19.79 ± 0.95	18.73 ± 0.39	17.61 ± 0.87	16.98 ± 0.55
ICA10	19.88 ± 0.91	19.92 ± 0.49	18.88 ± 0.74	17.78 ± 0.76	16.88 ± 0.76
ICA20	19.65 ± 0.87	19.84 ± 0.79	18.95 ± 0.77	18.11 ± 0.74∗	17.45 ± 0.81∗#

Data was expressed as mean ± SD. ∗*p* < 0.05 vs. NS group; #*p* < 0.05 vs. ZOL group. NS: the blank bone metastasis model group; ZOL: the zoledronic acid + bone metastasis group; ICA20: icariin 20 mg/kg + bone metastasis group; ICA10: icariin 10 mg/kg + bone metastasis group.

## Data Availability

The data used to support the findings of this study are available from the corresponding author upon request.
